This article has been retracted.

# Innovation and Exploration of Computer-Aided New Media Translation Course Teaching Mode under the Ecological Environment

**DOI:** 10.1155/2022/6305590

**Published:** 2022-10-10

**Authors:** Wei Zhou, Bei Gao

**Affiliations:** ^1^School of Foreign Studies, Harbin Engineering University, Harbin 150001, China; ^2^Department of Foundational Courses Teaching, East University of Heilongjiang, Harbin 150066, China

## Abstract

In order to analyze the innovation of computer new media-aided translation course teaching mode under the ecological environment, this paper introduces the CorpTrans system, which analyzes the practical effect of computer-aided translation system applied in the course teaching, verifies the role of the system in computer-aided translation course teaching, and plays an important role in improving students' translation ability. At the same time, starting with the development trend of new media environment, the CorpTrans system is used to innovate the teaching mode of computer-aided translation course. The teaching ecology of the comprehensive new media translation curriculum consists of the interaction between the ecological subject of teaching and the ecological environment of teaching. Through the efforts of both teachers and students, high-quality computer-aided translation courses will contribute to cultivating compound translation talents. The innovation of teaching mode needs to be realized by this system, so as to better meet the requirements of improving the teaching level of translation courses.

## 1. Introduction

From the perspective of ecology, the teaching process of comprehensive English curriculum is regarded as a teaching ecosystem, the application of corresponding new media in the process of comprehensive English curriculum teaching is discussed, and the relationship between new media technology and translation curriculum teaching is analyzed with ecological view. Computer-assisted translation is human-machine collaboration. As a tool to assist translators, computers can help translators improve performance, improve translators, simplify translation processes, and get more recycling. As shown in Figure 1, memory translation is an important part of computer-assisted translation.

Memory translations start with drawing and become “smarter” and get better as they learn and memorize. In addition, translation memories can identify the integration and integration of language tools and processes, playing an important role in managing models such as translation projects [1]. Keywords are words or terms selected from reports and papers for the purpose of document indexing to express the topic content information of the full text, which can clearly and intuitively express the literature discussion or reflect the theme of the article. Therefore, starting with keywords is a shortcut to quickly track the research status of a certain field. The classroom teaching ecological environment includes the following ecological factors: teaching materials, natural environment of the classroom, teaching media environment, teachers' ‘teaching literacy, and students' knowledge and skill literacy. After-class learning ecological environment involves the following ecological factors: the form and content of homework, students' ability of independent review and knowledge transfer, the media environment to assist learning, and the evaluation and assessment system of learning completion effect. The development trend of related research was examined based on keywords, and it was not hard to find that the research of this field presented an upward trend with slow speed in the past 15 years. Therefore, from the end of the last century to the beginning of this century, there were few researches on computer-aided interpretation teaching. And accompanied by small fluctuations, then it developed slowly, which showed a large growth after 2009 [2]. Although the attention of foreign language teaching and research circles in China is increasing day by day, the number of researches is still relatively small, and more investigations are still needed on the combination of computer and interpretation teaching in the emerging translation discipline.  Table 1 is the statistical analysis results based on the CNKI's measurement visualization analysis tools [3]. At the level of CAI research, 52.2% of them are basic researches, mainly focusing on Chinese language, foreign language, and computer software and its application. Translation is a common means of language transformation. Traditional translation only needs to express the general meaning of the article. Ecological translation, on the basis of translation, is a detailed interpretation of the translated work, starting from the ecological structure of the translated article, and keeps the meaning of the original sentence as much as possible in the process of translation. Ecological translation pays attention to the inherent ecological structure of translation language, which has certain translation characteristics.

“Mutualism” is one of the embodiments of the relationship between organisms in ecology, which refers to the mutual favorable relationship between the two species, and there is an interdependence between each other. “Computer-aided translation” is a keyword often used in the investigation of the research results of relevant course teaching, with computer-aided translation as the main direction. It can be seen that after dividing computer-aided translation into technical terms such as instruction and technology, “translator” and “teaching translator” are the basis of CAT research [4]. Among them, “translation guidance” includes “interpretation” and “classroom setting”. “Translator” connects the two values associated with the relationship, “translation memory” and “corpus”, and is the basis for the output of CAT technology. The two central nodes have crossover nodes such as “translation software” and “translation technology”, and these crossover nodes extend to peripheral nodes in specific application fields such as “localization”, “translation ability”, and “glossary” [5]. Tables 2 and 3 are the keyword frequency tables based on teaching and technical research topics, respectively. Combined with the previous analysis of computer-aided translation courses, it can be seen that the research of computer-aided translation in China started relatively late and began to develop formally in the 1980s. However, in the past decades, China has achieved exceptionally fruitful research results in this field [6]. With the development of cloud computing, artificial intelligence and other new computer technologies, the deepening of interdisciplinary research as well as the cooperation between insiders and academics, it is believed that the research of CAT in China will be more mature in the new development stage. Ecological factors refer to the environmental factors that directly or indirectly affect the growth, development, reproduction, behavior, and distribution of living organisms. In other words, all environmental factors outside the organism can be called environmental factors.

With the increasingly extensive communication in various countries, ecological translation has received more and more attention. From the perspective of ecological translation, teachers should give full play to the function and role of computer-assisted translation, focus on improving the accuracy of students' translation, and stimulate students' interest in learning this subject. Translation is a major that combines theory and practice, especially computer-aided translation. Computer-aided translation is also a course that combines knowledge and skills. Combining three-dimensional teaching objectives: methods and processes, knowledge and skills as well as emotional attitudes and values, it is also a course that focuses on knowledge and skills. In addition to learning the theoretical knowledge of computer-aided translation, students should also acquire the knowledge and skills related to translation [7]. Only when students possess and master certain knowledge, can complete translation work, and only when they are skilled enough in relevant skills, they can give full play to the role of computer-aided translation software. As a new technology, computer-aided translation is facing many opportunities and challenges in its development. High-quality computer-aided translation courses will play an important role in cultivating versatile translation talents. As the main training base of translation talents, colleges and universities are faced with difficulties such as monotonous teaching mode, outdated content, unideal ecological translation environment, and not prominent translator central position in the process of teaching implementation. In recent years, the vigorous development of ecology has provided a new theoretical perspective for language teaching and research and accelerated the pace of foreign language teaching reform in China.

## 2. Literature Review

Paying attention to the characteristics and functions of different environmental factors in ecology and adjusting and utilizing them can promote the teaching activities and literacy ability related to teaching subjects, such as the application of new media in the teaching of new media translation courses. Translation is the process of converting one language into another using a computer. The software used to do this is called a translator [8]. It is a borderline subject that studies how to use computers to carry out translation between natural languages and its effectiveness depends on human's general understanding of the expression mechanism of natural language and the operability of computer language translation [9]. Guarin et al. carried out the experiment of machine dictionary lookup, and the understanding of MT was still limited to word-to-word translation at that time [10]. Rule-based approach has long been the mainstream approach in machine translation research both at home and abroad. Through the understanding and induction of language phenomena, RBMT summarized its laws and formed a specific language grammar system. And on the basis of the grammar system, the input language was analyzed and understood, forming the unambiguous internal representation of language. The target translation was generated from the corresponding target language structure generated by this transformation [11]. From the perspective of reasoning mechanism, BRMT was a rationalist machine translation method. With the development and progress of computer software and hardware technologies, theories and technologies of artificial intelligence and computational linguistics, machine translation methods, and technologies were greatly improved and developed, and various machine translation methods made significant contributions to solving language barriers [12]. However, there were essential differences between computer and human brain. Due to the complexity and irregularities of natural language expression and the limitations of various machine translation methods, although workers on linguistics and computer experts came up with many methods, such as using computer simulation of the human brain function and ways of thinking, they always could not simulate the human beings' thinking [13]. In this context, ecological linguistics, as an interdisciplinary discipline, has emerged quietly. It mainly studies the interrelationship between language and ecological environment and advocates the study of the influence of environment on language from the perspective of ecology. The research topics include language acquisition, language survival, language diversity, language evolution, and language teaching. Therefore, so far, the translation quality and accuracy rate of machine translation system was still unsatisfactory, which could not achieve the degree of “faithfulness, expressiveness and elegance”.

## 3. Methods

These new media belong to the ecological environment in the ecosystem and can be regarded as the information media environment in the abiotic environment. These new media tools are applied to the auxiliary course teaching, and combined with the basic principles of ecological subject and environment-related in ecology, the characteristics and functions of new media as one of the environmental factors in the auxiliary course teaching ecology in the information media environment are analyzed. Translation memory technology can help us solve many practical problems, especially the sentences in the process documents in the field of mechanical manufacturing, which can reduce the amount of repeated labor, unify terms, and make the translation style tend to be consistent. However, it has never been realized in the field of mechanical manufacturing. And some key technologies involved in translation memory need to be further studied. There are many parables in the example library, which can be used as models for future translations [14]. In order to select similar example sentences, it is necessary to determine which example sentences in the instance library can be used to translate the input sentence to be translated, that is, it is necessary to determine the similarity between the sentence to be translated and the example sentences (namely similarity). So it is necessary to establish a set of corresponding similarity criteria. Although there are many theoretical researches on similarity, it is generally calculated by distance-based method in practice. And a detailed tree adverbial thesaurus is mainly relied on in the calculation process [15]. The training program and curriculum are completely formulated by the school, and the personal wishes of the learners are not fully considered. Ecological linguistics theory requires language teaching to learners as the center, students as the main body of learning, therefore, translation teaching should fully consider the learners' personal factors and related social and cultural factors, including learning methods, learning attitude, and expectations to find appropriate teaching methods and to gradually guide and implement the teaching. Some systems use simple methods as the only way to display information and do not take full advantage of the rich information in the semantic lexicon. The formula is as follows:

(1) $$\begin{array}{c} S=\frac{2\times i}{m+n}\times 100\%. \end{array}$$

In the formula, *S* is similarity degree, *i* is the number of the same words in the sentence to be translated as the example sentence, *m* is the total number of all words in the sentence to be translated, and *n* is the total number of all words in the example sentence.

If the ID string of the sentence to be translated is exactly the same as the ID string of the example sentence, that is, the overall similarity of the ID string is 100%, but the two sentences are not exactly the same, then the solution of the exact similarity needs to be fine-tuned within this range. This moderating similarity is called ID string fine-tuning similarity in the research [16]. Because ID string itself is the order number of each Chinese word, so each number is the only representative of the Chinese words and different parts of the string are only English. So the main task is to compare whether the English string is consistent or not. If they are completely consistent, then fine-tuning similarity of ID string is 100 at this time. If they are not same, then the fine-tuning similarity of ID string is 0% at this time [17]. The fine-tuning similarity of ID string is adjusted by 1% in the exact similarity, that is, the weight coefficient is 0.01 (The weight coefficient here is selected according to the actual needs of the developed system after several tests as shown below). The process of language acquisition is accompanied by an active and creative “ecological learning environment” composed of multiple factors, and learners can directly perceive the meaning of language when they are active in this environment. The “translator-centered theory” in the ecological translation theory is to regard the translator as an independent subject with creativity, sensibility, and leading role, and it is the cornerstone of making the whole translation process proceed continuously.

(2) $$\begin{array}{c} D_{w1}=\frac{n-m_{1}}{n}\times 100\%. \end{array}$$

In the formula, *D*_*w*1_ represents the fine-tuning similarity of ID string. *m*_1_ represents the total number of different English words in the sentence and *n* represents the total number of words in the sentence.

The fine-tuning similarity of ID string plus the overall similarity of ID string is the exact similarity of the final solution, namely:

(3) $$\begin{array}{c} D_{1}=D_{z1}+q_{z1}+D_{w1}+q_{w1}. \end{array}$$

In the formula, *D*_1_ stands for exact similarity. *D*_*Z*1_ represents the overall similarity of ID string. *q*_*z*1_ represents the weight coefficient of the overall similarity of ID string in the exact similarity, which is 0.99 in the research. *q*_*w*1_ represents the weight coefficient of the fine-tuning similarity of ID string in the exact similarity and the value is 0.01 in the research [18].

If the part-of-speech substring of the sentence to be translated is exactly the same as the part-of-speech substring of the example sentence, that is, the overall similarity of the part-of-speech is 100, while the ID strings of the two sentences are not exactly the same, fine-tuning is needed to solve the exact similarity. This moderating similarity is called the part-of-speech substring fine-tuning similarity in the research. Since the part-of-speech substring itself identifies the part-of-speech and part-of-speech substring of each word, the task of fine-tuning the similarity of the part-of-speech substring is to compare whether the numbers of each pair of words are consistent [19]. This translation teaching mode artificially split the translation integrity and relevance and destroyed the students' ‘“translation ecological environment”. The students' thinking and vision were greatly limited, it is difficult to effectively mobilize their learning enthusiasm and creativity, and their translation ability naturally cannot improve accordingly, thus they cannot adapt to the needs of the real society. If all the corresponding words between the sentences are to be translated, and the example sentences are exactly the same, then the fine-tuning similarity of the part-of-speech sub-string is 100%. If they are all different, then the part-of-speech substring fine-tuning similarity is 0%. The fine-tuning similarity of part-of-speech substring is adjusted 20% in the exact similarity, that is, the weight coefficient is 0.2.

(4) $$\begin{array}{c} D_{w2}=\frac{n-m_{2}}{n}\times 100\%. \end{array}$$

In the formula, *D*_*w*2_ represents fine-tuning similarity of part-of-speech substring. *m*_2_ represents the total number of words with different numbers in sentences except for English strings and *n* represents the total number of words in sentences.

The exact similarity of the final solution is shown as:

(5) $$\begin{array}{c} D_{2}=D_{z2}\times q_{z2}+D_{w2}\times q_{w2}+D_{w1}\times q_{w1}. \end{array}$$

In the formula, *D*_2_ represents exact similarity. *D*_*z*2_ stands for the global similarity of the part-of-speech substring. *q*_*z*2_ represents the weight coefficient of the total similarity of the part-of-speech substring in the exact similarity, and its value in the research is 0.79. *q*_*w*2_ represents the weight coefficient of the total similarity of the part-of-speech substring in the exact similarity, and the value is 0.2 in the research [20].

If the part-of-speech string of the sentence to be translated is exactly the same as the part-of-speech string of the example sentence, that is, the overall similarity of the part-of-speech string is 100%, but the part-of-speech substring of the two sentences is not exactly the same, then the solution of the exact similarity needs some fine-tuning processing. This moderating similarity is called part-of-speech string fine-tuning similarity in the research. The part-of-speech string includes keywords and nonkeywords. And the constraint conditions of the key part-of-speech are the same as those of the part-of-speech substring, but nonkeywords are different. Since nonkeywords only give the part-of-speech in the part-of-speech string, but not the part-of-speech subclass, the task of the part-of-speech string fine-tuning similarity is to compare whether the part-of-speech subclass of each nonkeywords is consistent [21]. If the subclasses of each word in the sentence to be translated are exactly the same and the fine-tuning similarity of the part-of-speech string is 100%. If they are all different, then the fine-tuning similarity of the part-of-speech string is 0%. The fine-tuning similarity of part-of-speech string is adjusted 15% in the exact similarity, that is, the weight coefficient is 0.15.

(6) $$\begin{array}{c} D_{w3}=\frac{n-m_{3}}{n}\times 100\%. \end{array}$$

In the formula, *D*_*w*3_ represents the fine-tuning similarity of part-of-speech subclasses. *m*_3_ represents the total number of words with different part-of-speech subclasses in the sentence, and *n* represents the total number of words in the sentence. In this ecological teaching mode, students are not only the main body of learning but also the main carrier of language acquisition and development. Therefore, the focus of teaching implementation is to make students realize their own translation ability and improve the degree of efforts. Of course, teachers are not only the organizer of classroom teaching and the instructor of the translation process but also the readers and judges of students' translation. “Translator-centered” does not mean denying the positive role of teachers.

No matter in Europe, America, or China, the dominant technique in machine translation has always been rule-based transformation. Rule-based machine translation is the most mature and widely used technology. This approach requires that knowledge about source and target languages be expressed in a form that computers can “understand”. The series of processes is the process of using the theory of artificial intelligence to establish the system and inference machine to imitate human brain translation [22]. The following terms are commonly used. Through his connection and understanding of common sense, he regularly writes his own rules, developing his own grammatical and semantic rules. The system uses these rules to identify entries, create internal proxies, and translate internal proxies to the target language to create translations.  Figure 2 is a general overview of a rights-based translator.

According to ecological theory, the environment in an ecosystem is a source of information. In the system, there is information transmission among the components, which is one of the basic functions of the ecosystem. The so-called “similarity” is a very vague concept, where there is no unified measurement standard. At present, there are many researches on similarity criterion abroad, but the specific application may be different in different systems. And all methods have one purpose, which is to judge the distance between the two words. All of these methods are based on calculating the similarity between words. In terms of overall structure, laws are mainly summarized from the general characteristics of each word in the sentence to be translated, such as the part-of-speech, part-of-speech subclass, and sequence number, and similar example sentences are preliminarily extracted from the sample sentences database by using these laws [23]. The emerging ecological language teaching concept creatively integrates the ecological theory with the language teaching process, attaches importance to the interaction relationship between the various elements of language learning, and emphasizes the relevant social and cultural factors, which has a strong advantage of cultural dependence and dynamic and unified and sustainable development. In the research, the similarity between sentences to be translated and example sentences on the whole is called global similarity. Example sentences are retrieved preliminarily according to the general similar structure. The similarities and differences of the sentences to be translated and example sentences are compared mainly in the part-of-speech, semantic, and so on, and the similarity degree of the two sentences on the vocabulary is shown. The lexical similarity between sentences to be translated and example sentences is called fine-tuning similarity.  Figure 3 shows the overall flow designed based on overall similarity and fine-tuning similarity.

After calculating the similarity of computer translation system, it is needed to clarify the two basic tools used in CorpTrans software design. The particularity of translation teaching requires the selection of flexible and effective teaching methods in the process of teaching implementation, paying attention to cultivating students' cross-cultural awareness and independent learning ability, and designing a teaching evaluation mechanism in line with students' expectations, so as to create an independent learning environment for learners and promote the benign interaction between teachers and students.

Work research method is through undertaking scientific analysis and determination to working method, working flow and working time, scientific and reasonable working standard, and time norm are worked out accordingly to make each work standardized and raise labor productivity and economic benefit ceaselessly. Work research is the most important basic technology in IE theory system. Its significance is that the future of the system can exceed the reality and improve productivity in the case of little or no investment [24]. From the perspective of ecology, respecting the law of language development and studying the various elements of language learning and the dynamic interaction between teachers and students can help to stimulate learners' interest in learning, improve their translation ability, and form translation thinking. This 5-level design method was also applied to the development of CorpTrans software, as shown in Table 4.

CorpTrans still takes into account the fact that traditional machine-aided translation is based on sentence pairs. because translating is the easiest when sentence level matching is achieved immediately. On this basis, the system will also adopt an auxiliary translation strategy below the sentence level, namely, block translation matching. So block level alignment is provided when sentence level matching is not possible, so as to provide more translation instances for users to choose and use. The matching term is divided into two parts: continuous term and noncontinuous sentence. Work researches were initially used to improve operating procedures for workers in machining workshops. Later, this method was transplanted to the service industry and gained great benefits. It was found that this classical method of industrial engineering was also very suitable for the compilation of translation software, which could greatly improve the efficiency and quality of targeted translation. Ecological theory believes that ecological balance means that the input and output of ecosystems tend to be equal over a long period of time, its structure and function are in a stable state for a long time, and it has the self-repair ability to cope with interference. So the ecological balance means that there must be a balance between living organisms and the environment. The latter creates another opportunity for the user to align at the sentence level by adding the corresponding term to the sentence structure after selecting it as shown in Figure 4.

Computer-aided translation software is mainly composed of memory bank, term bank, and word processing interface. The former two can achieve the effect of reusing the existing translation by matching the original text in the database, while the word processing interface undertakes the editing function. In order to achieve fast deployment, fast use, fast effect, and fast update, no matter in the architecture layer or the code level, the system should follow the principle of simplicity, keep a cautious attitude to add functions and eliminate the shackles of redundant functions. There should be fewer levels of data exchange and functional stratification in the system architecture, so as to meet the requirements of simplicity and improve the robustness of lightweight web applications. The flow chart of the system is shown in Figure 5. Under the influence of the foreign environment, the ecological balance needs to be realized by the self-regulation of the ecosystem, and the self-regulation depends on the feedback mechanism of the system. Therefore, in the teaching ecosystem, the application of various relevant new media in computer-aided course teaching should combine the teaching objectives and teaching objects as well as the characteristics and functions of the corresponding new media.

According to the system flow chart, four main modules can be divided into and designed:

1. *User Management Module*. It is the module that creates and manages the translators' account
2. *Project Management Module*. It is responsible for processing and importing the project from the .lang file, and providing users with project information as well as editing core function entries
3. *Term Management Module*. It is responsible for the implementation of term database and related operations, including term adding, term editing, and term detection tips
4. *Finished Product Project Publishing Module*. It exports the edited project to the finished product .lang file

Figure 6 shows the structural relationship between system functional modules.

The test module design of translation course is mainly to test the relevant knowledge points after students learn auxiliary translation tools. Specifically, teachers will select questions by random sampling after entering the question bank and then give them to students. After entering the interface, students can choose whether to take the test of aided translation course. If the examination is adopted, paper will be resubmitted to the system after the completion of the examination, and the examination ends. The teacher corrects the test papers and finally uploads the results to the system for students to query as shown in Figure 7.Coordinate the relationship between translation teaching and students' interests and social needs, and make full use of the modern network information platform, make full use of online, offline, class and off-class translation resources, combine theory with practice, and jointly create a harmonious “translation ecological environment”.

## 4. Results

As a component factor in the development of The Times, education naturally cannot develop independently from other ecological factors; so does the teaching of specific professional courses. In the research of CAT techniques and tools, the research procedures based on rules, subjects, and statistics are mature, but not deep enough. First, the grammatical and semantic models of Chinese are more complex than those of English, and the benefits of English studies cannot solve all problems. Scientists still need more attempts to determine China's uniqueness. Second, with the improvement of my country's economic cooperation level, the trade between mainland China and other countries in the world has increased, and the demand for services in small languages has increased a lot. The construction of bilingual and multilingual CAT translation platforms for ethnic minority languages has increasingly become the research object of major ethnic colleges and universities. However, due to social and historical reasons, such corpus is relatively lacking. And the construction and improvement of CAT corpus for ethnic minority languages will be a long-term process [25]. In our country, the demand for translation talents is expanding and improving today. The application of ecological theory into the specific translation teaching field and to reexamine the problems existing in the translation teaching process of the universities in our country are conducive to build a harmonious ecological translation teaching mode, improve the quality of translation teaching for the country and society to cultivate high-level, professional, compound foreign language talents. Thirdly, CAT technology tools are mainly based on text processing, and there are few researches on speech. At present, IFLYTEK has made a major breakthrough in the field of language recognition. The similarity calculation method based on distance is used to calculate the similarity of translated sentences and Chinese example sentences at sentence level and lexical level, respectively, by using the similarity calculation method based on overall similarity and fine-tuning similarity. The implementation of computer-aided translation system with translation memory technology as the core in the field of aircraft manufacturing has significantly reduced the workload of translation. Because of the guarantee of the unity of terms and the repeated use of translation results, the style of translated versions is basically the same, and the use of terms does not conflict. The research on memory translation device and computer-aided translation knowledge can meet the goals of product development and practical application and has achieved certain results. According to the application of translation software, in order to improve the teaching efficiency of computer translation services under new media, teachers need to improve their professional knowledge and skills, attention, and relationship between teachers and students. The appropriate difficulty of the translation of the original text should be selected to maintain students' moderate learning motivation. It is difficult to combine computer course with other courses. In order to provide high-quality courses, it is necessary to improve the relevant knowledge of this course, especially to continuously investigate the principles, terms, corpus, and other knowledge of computer translation software. When explaining how to make corpus and other practical operations, teachers should keep in mind the steps of this operation. Before the class, students should be prepared to meet the problems. In class, teachers should do a good job of guiding students to operate in reality. After class, teachers should do a good record and teaching reflection. Teachers need to adopt a certain educational mechanism to pay attention to the status of students and adopt effective interactive methods, so as to establish a good teacher-student relationship. Computer-aided translation (CAT) courses are designed to help students to translate different texts using CAT software. Language is a tool for people to understand and transform the world. It is also an important carrier connecting the mutual relationship between people, people and society, and people and culture. In the field of foreign language teaching and research, the use of ecological principles and methods to study the law of the interaction between foreign language teaching activities and its external environment will provide a more comprehensive and systematic ecological perspective for translation teaching and research. Therefore, teachers should consider the difficulty of teaching according to their aptitude in the selection of texts and let students try to translate texts in different fields as much as possible. From the perspective of students, in the context of new media, students need to correct their learning attitude and build up their confidence in order to improve the teaching effect of computer-aided translation. Students should understand the importance of the course and believe that computer-aided translation software will be the inevitable trend of translation in the future. At the same time, it also alleviates the fear of liberal arts students on the curriculum. Students should be encouraged to learn in a variety of ways. The way of learning for college students should not only be limited to the classroom. Outside the classroom, students have enough time to control themselves. Students can learn, consolidate, and study CAI through self-study, studying with classmates, online learning, and other channels. Students should be guided to expand their knowledge and become qualified interpreters in the new era. For the language service industry, the primary basic quality of a qualified interpreter is to master a wide range of knowledge [26]. However, for most undergraduate students majoring in translation, they think that it is enough to learn professional knowledge and work hard to obtain professional certificates or pass the postgraduate entrance exam. Therefore, it is necessary to infiltrate the necessity of learning comprehensive knowledge into students and encourage them to read more books and read good books, so as to lay a solid foundation for future translation work.

## 5. Conclusion

From the perspective of ecology, its teaching subject, teaching object, teaching content, and teaching methods constitute a teaching ecosystem. This ecosystem involves ecological subjects, ecological and environmental factors, etc. In the new era of rapid development, the demand for talent in the translation market is increasing. And numerous manuscripts need to be completed efficiently and with high quality for translators. Human translators are limited to about 5,000 words a day. But with the help of computer-aided software, they can increase their workload to more than 10,000 words a day. Translators are no longer just good at translation, but those who not only translate but also have comprehensive knowledge and skills, which undoubtedly includes the use of computer-aided software to carry out translation work. In order to cultivate modern translation talents, more and more universities set up computer-aided translation courses, which cannot only train students to translate with translation tools but also promote the development of computer-aided software. As a new technology, CAT is facing many opportunities and challenges in the process of development. For both teachers and students, the importance of this course is self-evident. As a product of modern science and technology, new media is one of the many environmental factors affecting the stable development of the teaching ecosystem. This teaching ecosystem needs to maintain an ecological balance. Therefore, in the teaching process, it is necessary to view the influence of various new media tools on the whole teaching ecosystem to face the ecological function of new media and the ecological efficiency. However, in order to cultivate more translation talents in the translation industry, it needs to be based on computer-aided translation software. More specifically, these specific measures should be taken as follows:

1. Teachers should constantly improve themselves, adopt flexible teaching methods, attach importance to teacher-student relationship, and select appropriate translation original texts
2. Students are required to correct their learning attitude and have confidence in the course. In addition to the classroom learning, they should continue to learn computer-aided translation software and other comprehensive knowledge through self-study and cooperative learning

Students are not only the builders of knowledge but also the core of the teaching implementation process. The process of language acquisition is accompanied by an active and creative “ecological learning environment” composed of multiple factors. Through the efforts of both teachers and students, high-quality computer-aided translation courses will play an important role in cultivating versatile translation talents.

## Figures and Tables

**Figure 1:** Computer-aided translation.

**Figure 2:** General flow of rule-based machine translation.

**Figure 3:** General process of similarity solving problems.

**Figure 4:** CorpTrans system design process.

**Figure 5:** Another system flow chart.

**Figure 6:** System module design.

**Figure 7:** The implementation process of examination module.

**Table 1:** Statistics of retrieval results.

Keyword	Electronic brain-aided translation	Auxiliary machine translation	Machine-aided translation	Aided translation	Computer-aided translation	Total
The article number	1	10	18	23	579	631

**Table 2:** Statistics of the keyword frequency of teaching research topics.

Research topics	Keyword	Frequency	Total	Percentage
Teaching	CAT teaching	18	90	28.40%
	The curriculum	14		
	Translation teaching	34		
	Master of translation	11		
	Translation ability	13		

**Table 3:** Statistics of the keyword frequency of technical research topics.

Research topics	Keyword	Frequency	Total	Percentage
Technology	Translation memory	53	167	52.80%
	Glossary	11		
	Corpus	23		
	Machine translation	61		
	Translation techniques	19		

**Table 4:** System design level and content.

Presentation layer		Visual design	
Framework layer	Interface design		Navigation design
		Information design	
Structure layer	Interaction design		Information architecture
Scope layer	Function specification		Content demand
Strategy layer		User demand	
		System goals	

## Data Availability

The labeled data set used to support the findings of this study is available from the corresponding author upon request.
